# A Nomogram for Predicting Physical Restraint of Patients in Intensive Care Unit

**DOI:** 10.1155/2023/6618366

**Published:** 2023-04-17

**Authors:** Yun Wang, Ying Liu, Ya-Li Tian, Su-Lian Gu

**Affiliations:** ^1^Department of Geriatric ICU, Jiangsu Province Hospital, Nanjing, China; ^2^Department of ICU, Jiangsu Province Hospital, Nanjing, China; ^3^Department of Neurology ICU, Jiangsu Province Hospital, Nanjing, China

## Abstract

**Background:**

Despite its ethical implications, physical restraint (PR) is widely used in the intensive care unit (ICU) to guarantee the safety of patients. This study investigated the frequency and risk factors of PR use for patients in the ICU to establish a predictive nomogram.

**Methods:**

Clinical parameters of patients admitted to the ICU of Jiangsu Province Hospital from January 2021 to July 2021 were retrospectively collected. Independent risk factors of PR were analyzed by univariate and multivariate logistic regression analyses. The R software was used to establish the nomogram. Model performance was validated using the concordance-index (C-index) and calibration curves.

**Results:**

The rate of PR use was 46.32% (233/503 patients). Age (*B* = 0.036, odds ratio [OR]: 1.037, 95% confidence interval [CI]: 1.022–1.052, *P* < 0.001), consciousness disorder (*B* = 0.770, OR: 2.159, 95% CI: 1.216–3.832, *P*=0.009), coma (*B* = −1.666, OR: 0.189, 95% CI: 0.101–0.353, *P* < 0.001), passive activity (*B* = 1.014, OR: 2.756, 95% CI: 1.644–4.618, *P* < 0.001), delirium (*B* = 0.993, OR: 2.699, 95% CI: 1.097–6.642, *P*=0.031), −3 < Richmond Agitation Sedation Scale (RASS) score <2 (*B* = 0.698, OR: 2.009, 95% CI: 1.026–3.935, *P*=0.042), RASS score ≥2 (*B* = 1.253, OR: 3.499, 95% CI: 1.126–10.875, *P*=0.030), and mechanical ventilation (*B* = 1.696, OR: 5.455, 95% CI: 2.804–10.611, *P* < 0.001) were identified as independent risk factors for PR in the ICU (*P* < 0.05) and included in the nomogram. The C-index was 0.830, and the calibration curve indicated good discriminatory ability and accuracy (mean absolute error: 0.026).

**Conclusion:**

The prediction nomogram model of PR in ICU was established based on age, mobility, delirium, consciousness, RASS score, and mechanical ventilation. It showed good discrimination and accuracy. This nomogram may predict the probability of PR use in the ICU and guide nurses in developing precise interventions to reduce the rate of PR.

## 1. Introduction

Physical restraint (PR) refers to the use of any physical or mechanical equipment, material, or tools to limit the movement of an individual [1]. PR is commonly used in clinical practice worldwide, particularly in the intensive care unit (ICU). Patients in the ICU are in critical condition. Owing to the unfamiliar treatment environment, suffering associated with diseases, and particularity of treatment, patients often experience emotional instability and restlessness. Furthermore, they may be unable to control their behavior. For example, they may unintentionally remove important life support equipment, such as tracheal intubation, central venous catheter, or other drainage tubes [2]. Therefore, PR is often applied to protect patients from the risk of falls and displacement of invasive devices due to irritability or delirium, which may result in treatment disruption [3, 4].

Numerous studies have reported that the percentage of patients subjected to PR in the ICU ranges from 32.9% to 76.0% [5–7]. In China, this percentage ranges from 38.8% to 80.5% [8, 9]. However, inappropriate use of PR may result in adverse events, which should be taken into consideration by nurses. Improper restraints can result in detrimental physical and psychological consequences (e.g., skin injuries, tissue injury, and delirium), which may even lead to post-traumatic stress disorder, asphyxia, and death [10–12]. Therefore, in order to guarantee patients' safety, it is crucial to minimize the pain experienced by them and reduce the rate of PR. Currently, in clinical work, adoption of PR is mainly determined by nurses according to their experience, which is more or less subjective. Hurlock-Chorostecki and Kielb [13] reported that a simplified clinical decision support tool helped critical care nurses make decisions about the use of restraints. However, nurses will use a clinical decision support tool but will forgo the recommendation of the tool to prevent disruption of treatment devices [14]. So, more decision-making tools are needed to reduce the PR use.

For this purpose, it is essential to understand the current status of PR for ICU patients and to identify influencing factors. Such knowledge would allow the development of effective strategies and guidelines to reduce the use of PR. The objectives of this study were to analyze the status of PR use among patients in the ICU, identify potential factors influencing the use of PR, and establish a nomogram for predicting the risk of PR use. Thereby, theoretical basis for formulating targeted interventions in ICU practices can be provided. The prediction model will provide supporting evidence to identify high-risk patients with PR and intervene in advance, which can help nurses make decisions about PR, and thus reduce the rate of PR.

## 2. Materials and Methods

### 2.1. Study Subjects

In this retrospective study, we collected data of patients who were hospitalized in the ICU at Jiangsu Province Hospital (Nanjing, China) from January 2021 to July 2021. Patients were divided into the PR and non-PR groups based on the use of restraint during hospitalization. The inclusion criteria were age ≥18 years; ICU stay ≥24 h; and availability of complete data in the electronic records system. Patients with a history of mental illness and those in close or protective isolation were excluded from this analysis.

### 2.2. Sample Size Calculation

Based on a literature search, 13 potential factors were preliminarily included in this study. As a rule of thumb, there shall be at least 10 events per candidate variable for the derivation of a model. According to the statistics in Jiangsu Province Hospital, the rate of PR for ICU patients in 2020 was 31.14%. Assuming a 10% rate of invalid cases, the formula for calculation is as follows. Therefore, the target population for inclusion in this study was 503 patients.

(1) $$\begin{array}{c} n=\frac{\text{Number of variable}\times 10}{\text{Rate of physical restraint}\times \left(1-10\%\right)}\text{.} \end{array}$$

### 2.3. Data Extraction

Data extraction was conducted in the ICU by two of our investigators after uniform training. They checked the data together to ensure the data accuracy. Medical and nursing electronic records were reviewed to collect patients' data. Demographic and clinical data were collected. Data on the following variables were extracted: sex; age (years); body mass index (BMI); disease classification; consciousness; activity ability; Richmond Agitation Sedation Scale (RASS) score; delirium; muscle strength; high-risk tubes; use of mechanical ventilation; use of sedatives; and use of analgesics.

### 2.4. Model Construction and Validation

Data analysis was performed to identify variables significantly associated with PR use. Variables which exhibited statistical significance in the univariate analysis were included in the multivariate regression analysis for the stepwise identification of independent predictors and development of a predictive model. The nomogram was established using the R software. The concordance-index (C-index) and calibration curves were used to evaluate the performance of the model.

### 2.5. Statistical Analysis

Data were analyzed by the SPSS version 23.0 (IBM Corp., Armonk, NY, USA) and R version 4.1.0 software (R Foundation for Statistical Computing, Vienna, Austria). Continuous variables with normal distribution were expressed as mean ± standard deviations, while non-normally distributed continuous variables were expressed as the median and interquartile range. These variables were compared using *t*-tests or the Mann–Whitney *U* test, in which *t* or *Z* statistics were used. Categorical variables were expressed as numbers and percentages. These variables were compared by the chi-squared or Fisher's exact tests, in which *χ*^2^ statistic or *P* value was used. Univariate analysis was used to identify variables significantly associated with PR. Forward elimination was employed to select the final set of risk factors independently associated with PR. A predictive nomogram model was established according to the regression coefficient of the final variable. The nomogram was established using the “rms” package. Calibration curves based on 1,000 bootstrap resampling iterations were used to examine the performance of the nomogram (internal validation). The C-index was used to assess the predictive ability of the nomogram. A *P* value of <0.05 denoted statistically significant difference.

## 3. Results

### 3.1. Univariate Analysis of Risk Factors Influencing PR

A total of 503 patients (323 males and 180 females) were included in this study. Among those, 233 patients (46.32%) were subjected to PR. The average age was 66.92 (standard deviation: 16.17) years, and the average BMI was 22.17 (standard deviation: 3.59). Univariate analysis revealed that age (*Z* = −5.389, *P* < 0.001), consciousness (*χ*^2^ = 27.129, *P* < 0.001), activity ability (*χ*^2^ = 37.110, *P* < 0.001), delirium (*χ*^2^ = 30.642, *P* < 0.001), use of analgesics (*χ*^2^ = 6.927, *P*=0.008), use of sedatives (*χ*^2^ = 4.008, *P*=0.045), use of mechanical ventilation (*χ*^2^ = 43.111, *P* < 0.001), RASS score (*χ*^2^ = 26.053, *P* < 0.001), and high-risk tubes (*χ*^2^ = 19.734, *P* < 0.001) differed significantly between the PR and non-PR groups (Table 1).

### 3.2. Multivariate Analysis of Risk Factors Influencing PR

The multivariate logistic regression analysis revealed that the following variables were significantly associated with PR use: age (*B* = 0.036, OR: 1.037, 95% CI: 1.022–1.052, *P* < 0.001); consciousness disorder (*B* = 0.770, OR: 2.159, 95% CI: 1.216–3.832, *P*=0.009); coma (*B* = −1.666, OR: 0.189, 95% CI: 0.101–0.353, *P* < 0.001); passive activity (*B* = 1.014, OR: 2.756, 95% CI: 1.644–4.618, *P* < 0.001); delirium (*B* = 0.993, OR: 2.699, 95% CI: 1.097–6.642, *P*=0.031); −3 < RASS score < 2 (*B* = 0.698, OR: 2.009, 95% CI: 1.026–3.935, *P*=0.042); RASS score ≥2 (*B* = 1.253, OR: 3.499, 95% CI: 1.126–10.875, *P*=0.030); and mechanical ventilation (*B* = 1.696, OR: 5.455, 95% CI: 2.804–10.611, *P* < 0.001). Notably, coma was a protective factor for PR (Table 2).

### 3.3. Nomogram Construction and Validation

A nomogram incorporating age, consciousness, activity ability, RASS score, delirium, and mechanical ventilation was established (Figure 1). The calibration curve indicated that the predicted probabilities by the nomogram fitted extremely well with the actual data (Figure 2). The model exhibited a C-index of 0.830, which suggested that the prediction model had good discriminatory and predictive ability.

## 4. Discussion

ICU patients' condition accompanied by varying degrees of consciousness disorder and irritability is critical, which may render their unconscious withdraw of lines such as vascular access or tracheal intubation. Furthermore, their unconscious behavior may endanger their lives. In order to prevent the patients from injuring others or themselves and guarantee progress of treatment, nurses usually apply PR on patients. In this study, the rate of PR among patients in the ICU was 46.32%, which is similar to those previously reported [15, 16]. However, Zhang et al. [17] reported that this rate may be as high as 59.07%. According to a survey involving 34 ICUs in Europe, PR was not utilized in two ICUs in Turkey and four ICUs in the United Kingdom [18]. Therefore, it is possible to reduce or even avoid the use of PR in the ICU. In 2017, the Joanna Briggs Institute Evidence-based Health Care Centre [19] proposed to reduce the use of PR and conduct a comprehensive evaluation of patients before PR application. These recommendations aimed at preventing the occurrence of adverse events associated with PR. This is particularly important in the field of clinical nursing.

As shown in this study, patients who were older and with consciousness disorder were subjected to PR more frequently than other patients. Comatose patients were less likely to be restrained. This finding supports the results of previous reports which revealed that age and consciousness were factors related to the use of PR [16, 20]. The population of China is gradually aging; hence, patients admitted to the ICU also tend to be older. The physical and cognitive functions of individuals deteriorate with increasing age. Moreover, older individuals are at an enhanced risk of falling from bed and self-injury. Restraint can be used to prevent such accidents [21]. Patients with consciousness disorder are characterized by poor communicating and cooperating ability, which are occasionally accompanied by agitation and disorientation. Hence, protective restraint is generally utilized in such patients to prevent self-injury or other injuries. In contrast, patients with coma or deep sedation are in a passive state of treatment and have a low risk of accidental extubation or falling from bed [22].

In this study, the probability of PR in patients with passive activity was 2.756-fold higher than that of patients with active activity. Patients with active activity are often conscious, as well as they can communicate and cooperate. However, patients with passive activity are characterized by poor ability for cooperation and are at a high risk of extubation or falling from bed. In addition, nurses may be unaware of the changing conditions of patients and have poor knowledge of indications for PR use, thereby resulting in more frequent restraint of passive patients. The decision-making process for the application of PR in the ICU is complicated and influenced by patients and their families, nurses, and management factors [23]. However, most nurses have poor knowledge regarding PR and insufficient practical experience [24]. Currently, there is a lack of assessment tools for PR. Therefore, an accurate predictive model can assist nurses in this setting. In addition, intervention measures can be taken in advance, which can reduce the use of PR.

In this study, delirium and RASS score were identified as independent factors related to PR use. This is consistent with the findings of previous studies [5, 25, 26], which described delirium and sedative drugs as the main factors linked to the use of PR in patients. It has been demonstrated that approximately one-third of patients in the ICU experience delirium [27] and frequently suffer altered mental status, poor concentration, confusion, or altered level of consciousness [28]. Due to perceived and actual risk enhancement of line removal or self-harm, ICU patients are often restrained once they develop delirium [11]. In this study, 16.70% of the patients experienced delirium, and 73.81% of those had been restrained. However, numerous studies have found that the use of PR is closely related to the occurrence and development of delirium. Moreover, PR and delirium can lead to a vicious circle [29, 30]. Therefore, medical staff should pay attention to the applicability of PR to patients with delirium for active prevention and treatment. In addition, medical staff should take alternative restraint methods to reduce the potential harm caused by PR in patients with delirium if necessary.

Owing to the common use of sedative medicines in ICU patients, this factor did not independently influence the application of PR in this study. Furthermore, influence of sedative medicines on PR also depends on the type, dosage, and degree of sedation. The present study demonstrated that patients with a −3 < RASS score < 2 were at a 2.009-fold higher risk of being physically restrained versus those with a RASS score ≤ −3. Patients with a RASS score ≥2 were at a 3.499-fold higher risk of being physically restrained than those with a RASS score ≤ −3. Moreover, PR was frequently applied to patients with a RASS score > −3. Patients with a RASS score ≤ −3 were in deep sedation, responding only to sound or physical stimuli. As for those patients, PR was not necessary [18].

In contrast, lightly sedated patients were more likely to experience agitation at any time; hence, nurses would restrain these patients in advance. Luk et al. [31] reported agitation (Sedation-Agitation Scale >4) as an influencing factor for PR; this finding is consistent with the results of this study. It is believed that agitated patients have poor ability for cooperation and were at risk of extubation or falling out of bed. Moreover, the ICU implemented an unaccompanied care system, thereby preventing family members from psychologically reassuring the patients. Moreover, the number of nursing personnel was not large enough for individualized care. Hence, nurses utilized PR to guarantee the safety of patients. Reasonable sedation, as well as timely and dynamic assessment of the extent of sedation, could help nurses make better restraint decisions and reduce PR use.

The use of mechanical ventilation, which was identified as an independent factor associated with PR use in this study, is directly related to patient survival. Previous studies have also reported mechanical ventilation as an independent associated factor [25]. Furthermore, a qualitative study of critical care nurses yielded results similar to that of this study. After nurses assessed patient awareness and behavior, they reported that PRs were the most protective methods of the endotracheal tube in critically ill patients (especially elderly patients), among whom the unplanned removal of medical devices was considered life-threatening [32]. A previous study demonstrated that tracheal intubation increased the risk of patients, who were physically restrained within 48 h after admission to the ICU [28]. In 2013, a study of 121 ICUs in France indicated that over 50% of mechanically ventilated patients experienced at least one PR. In addition, in 65% of ICUs, mechanically ventilated patients were restrained for more than half of the duration of mechanical ventilation [22]. Similarly, an online survey of 129 ICUs in Japan revealed that PR was frequently applied to mechanically ventilated patients in more than 40% of ICUs, and the proportion of those restrained was over 75% [33]. The incidence of unplanned extubation for tracheal intubation ranges from 3.0% to 22.1% [34, 35]. As for mechanically ventilated patients, the prevention of accidental extubation of tracheal tubes is vital for guaranteeing the patients' safety. Nonetheless, based on previous studies, unplanned extubation occurred among 25%–87% of patients during PR processes [36]. Numerous studies have even demonstrated that PR could increase the risk of unplanned extubation in patients [37]. With recent advancement of restraint reduction program, it can be found that a reasonable reduction in restraint could drastically reduce the incidence of unplanned extubation among patients with tracheal intubation [38, 39]. Therefore, PR may not prevent extubation in patients. Proper fixation, close observation, and timely assessment for tube retention are important measures to preclude unplanned extubation. These measures may improve the nursing quality offered to patients with mechanical ventilation, as well as patients with PR. To sum up, as for patients with mechanical ventilation, benefits and risks of PR use should be fully balanced in clinical practice.

The range of C-index is 0.5–1.0; higher values indicate better discriminatory ability of the model [40]. The BootStrap method was employed in this study to internally validate the predictive nomogram model for PR in ICU patients. The C-index of the nomogram was 0.830, indicating excellent discriminatory ability. The calibration curve of the nomogram showed an outstanding agreement between prediction and actuality. The actual probability with a mean absolute error of 0.026 indicated that this model was significantly accurate. Medical staff can use this nomogram to determine the risk of PR for each patient. Subsequently, targeted preventive measures and personalized nursing can be implemented to reduce the use of PR according to the influencing factors. For example, a 70-year-old patient with mechanical ventilation, disordered consciousness, and delirium, has a very high risk of PR according to the nomogram. Nurses can take measures of reasonable sedation, delirium treatment, and tube removal in advance to reduce PR use. The prediction nomogram model was more comprehensive than the restraint decision wheel which included behavior level, devices level, and independent level to determine when to use PR [13]. The nomogram addressed other factors that promote or inhibit device removal, such as the activity level, sedation level, or delirium.

Nevertheless, this study has the following limitations. Firstly, this was a single-centre retrospective study with a relatively small sample size. Thus, further validation by several multicentre and prospective studies is required. Secondly, although the nomogram exhibited good predictive ability, it is necessary to validate this model in the real world through a sequential prospective cohort study.

In summary, a predictive nomogram for PR was established for patients admitted to the ICU based on age, activity, delirium, consciousness, RASS score, and mechanical ventilation. The nomogram exhibited good discriminatory ability and accuracy. It can be used to rapidly predict the probability of PR among patients in the ICU and assist medical staff in identifying high-risk patients. Through this approach, preventive measures can be taken in advance to reduce PR use. Furthermore, the nomogram can help nurses make more objective decisions regarding PR use, avoid unnecessary or inappropriate PR, and take precautions to improve comfort of patients.

## Figures and Tables

**Figure 1:** Nomogram predicting the probability of physical restraint in the ICU. To use the nomogram, vertical line was drawn from each variable up to the point. The resulting value is the patient's score on that variable (i.e., “delirium = Yes” = 31 points). The scores for each variable were then summarized to obtain a total score corresponding to the risk of physical restraint. We then plotted a vertical line from the axis of the total point down to the risk of physical restraint, thus obtaining the physical restraint probability for this patient. ICU, intensive care unit; MV, mechanical ventilation; RASS, Richmond Agitation Sedation Scale.

**Figure 2:** Calibration curves of the nomogram. It showed that the predicted probabilities by the nomogram fitted extremely well with the actual data.

**Table 1:** Univariate analysis of physical restraint in ICU patients.

Factor	PR group (*n* = 233)	Non-PR group (*n* = 270)	*χ* ^2^ * /Z*	*P*
Age, years, median (IQR)	72 (63,83)	65 (54,74)	−5.389	<0.001
BMI, median (IQR)	22.490 (19.305, 24.650)	22.325 (19.530, 25.138)	−0.723	0.470
Sex, *n* (%)				
Male	147 (63.09)	176 (65.19)	0.239	0.625
Female	86 (36.91)	94 (34.81)		
Disease classification, *n* (%)				
Respiratory system	47 (20.17)	69 (25.56)	10.406	0.065
Digestive system	29 (12.45)	39 (14.44)		
Nervous system	42 (18.03)	43 (15.03)		
Circulatory system	34 (14.59)	28 (10.37)		
Postoperative	61 (26.18)	52 (19.26)		
Other	20 (8.58)	39 (14.44)		
Consciousness, *n* (%)				
Conscious	128 (54.94)	164 (60.74)	27.129	<0.001
Disorder	69 (29.61)	33 (12.22)		
Coma	36 (15.45)	73 (27.04)		
Activity ability, *n* (%)				
Active	58 (24.89)	139 (51.48)	37.110	<0.001
Passive	175 (75.11)	131 (48.52)		
Delirium, *n* (%)				
No	171 (73.39)	248 (91.85)	30.642	<0.001
Yes	62 (26.61)	22 (8.15)		
Analgesics, *n* (%)				
No	125 (53, 65)	176 (65.19)	6.927	0.008
Yes	108 (46.35)	94 (34.81)		
Sedatives, *n* (%)				
No	106 (45.49)	147 (54.44)	4.008	0.045
Yes	127 (54.51)	123 (45.56)		
Mechanical ventilation, *n* (%)				
No	100 (42.92)	194 (71.85)	43.111	<0.001
Yes	133 (57.08)	76 (28.15)		
RASS score, *n* (%)				
≤−3	28 (12.02)	62 (22.96)	26.053	<0.001
−3 < RASS < 2	161 (69.10)	192 (71.11)		
≥2	44 (18.88)	16 (5.93)		
Muscle strength, *n* (%)				
0–2	34 (14.60)	60 (22.22)	4.794	0.091
3	82 (35.19)	87 (32.22)		
4-5	117 (50.21)	123 (45.56)		
High-risk tubes, *n* (%)				
No	43 (18.45)	98 (36.30)	19.734	<0.001
Yes	190 (81.55)	172 (63.70)		

Note: BMI, body mass index; ICU, intensive care unit; IQR, interquartile range; PR, physical restraint; RASS, Richmond Agitation Sedation Scale.

**Table 2:** Logistic regression analysis of factors influencing the use of physical restraint.

Factor	B	SE	Wald	*P* value	OR (95% CI)
Age	0.036	0.007	23.913	<0.001	1.037 (1.022–1.052)
Consciousness	—	—	40.738	<0.001	—
Consciousness disorder	0.77	0.293	6.91	0.009	2.159 (1.216–3.832)
Coma	−1.666	0.319	27.324	<0.001	0.189 (0.101–0.353)
Passive activity	1.014	0.263	14.811	<0.001	2.756 (1.644–4.618)
Delirium	0.993	0.459	4.67	0.031	2.699 (1.097–6.642)
Analgesics	−0.225	0.265	0.718	0.397	0.799 (0.475–1.343)
Sedatives	0.153	0.292	0.276	0.599	1.166 (0.658–2.065)
Mechanical ventilation	1.696	0.34	24.968	<0.001	5.455 (2.804–10.611)
RASS score ≤ −3	—	—	6.264	0.044	—
−3 < RASS score < 2	0.698	0.343	4.139	0.042	2.009 (1.026–3.935)
RASS score ≥ 2	1.253	0.579	4.688	0.030	3.499 (1.126–10.875)
High-risk tubes	0.189	0.288	0.432	0.511	1.209 (0.687–2.127)
Intercept	−4.668	0.699	44.637	<0.001	0.009

Note: CI, confidence interval; OR, odds ratio; RASS, Richmond Agitation Sedation Scale; SE, standard error.

## Data Availability

All the data generated or analyzed during this study are included in this article. The processed data are available from the corresponding author upon reasonable request.
